The article "A Polylobar Nucleus Identifying and Extracting Method for Leukocyte Counting" was published in 2021. Journal: Comput Math Methods Med.

# A Polylobar Nucleus Identifying and Extracting Method for Leukocyte Counting

**DOI:** 10.1155/2021/5565156

**Published:** 2021-07-22

**Authors:** Jin Chen, Yiping Cao, Jie Gao, Haihua An

**Affiliations:** College of Electronic Information Engineering, Sichuan University, Chengdu, Sichuan 610064, China

## Abstract

Accurate counting of leukocytes is an important method for diagnosing human blood diseases. Because most nuclei of neutrophils and eosinophils are polylobar, it is easily confused with the unilobar nuclei in nucleus segmentation. Therefore, it is very essential to accurately identify and determine the polylobar leukocytes. In this paper, a polylobar nucleus identification and extracting method is proposed. Firstly, by using the Otsu threshold and area threshold method, the nuclei of leukocytes are accurately segmented. According to the morphological characteristics of polylobar leukocytes, the edges of the mitotic polylobar leukocytes are detected, and the numbers of polylobar leukocytes are determined according to the minimal distance rule. Therefore, the accurate counting of leukocytes can be realized. From the experimental results, we can see that using the Otsu method and the area threshold to segment the polylobar nuclear leukocytes, the segmentation ratio of the leukocyte nucleus reached 98.3%. After using the morphological features, the polylobar nuclear leukocytes can be accurately counted. The experimental results have verified the feasibility and practicability of the proposed method.

## 1. Introduction

In recent years, with the rapid development of computer science and digital image technology, biomedical image processing technology has emerged as a new interdisciplinary subject [1, 2] and has provided a reference for medical diagnosis and biological research [3, 4]. Biomedical engineering is closely related to related technologies such as Pattern Recogniton (PR) [5], Digital Image Processing (DIP) [6], Signal Processing (SP) [7], and Artificial Intelligence (AI) [8]. In biomedical imaging, the main technologies include laser microscopy and optical microscopy; in human medical imaging, the main technologies include CT, X-ray imaging, and electrocardiograms [9, 10]. The analysis and recognition of blood leukocyte images are widely used in biomedical image processing technology, and it is a complex and significant research topic [11–14]. The precise segmentation of blood leukocyte images is the most critical step, laying the foundation for subsequent analysis and classification research. At the same time, accurate counting of leukocytes is an important way of medical diagnosis [15–17]. Therefore, the segmentation and counting of leukocytes have become a research hotspot at home and abroad [18–20].

The article "A Polylobar Nucleus Identifying and Extracting Method for Leukocyte Counting" was published in 2021. Journal: Comput Math Methods Med.

To solve the problem of blood leukocyte segmentation, many kinds of segmentation schemes have been proposed. The image segmentation method based on geometrically deformable models [21, 22] can change the topological structure of the model while avoiding the high dependence on the initial contour, but the convergence speed is limited. Another proposed method is the image segmentation based on a genetic algorithm [23]. Although the genetic algorithm effectively solves the problem of getting into an infinite loop during iterative operations, the convergence is better. However, the genetic algorithm needs to encode the existing problems first, which increases the difficulty of the algorithm implementation. To solve the problem of leukocyte counting, W.H.Coulter achieves the automatic counting of particles based on the principle of electrical impedance [24]. However, this method leads to the problem that the blood sample cannot be preserved and the cleaning process of the instrument is complex. The number and types of leukocytes in the blood can reflect a person's health status [25], but most hospitals still take manual detection as the main method [26], and there are many shortcomings in manual detection. Different kinds of leukocytes play different roles in the human body and reflect different health states of the human body. In order to improve the accuracy and efficiency of leukocyte test and reduce the workload of medical staff, the accurate count of leukocytes is essential for the diagnosis of blood diseases.

Based on the complexity of blood leukocyte images, there are more polylobar nuclei in eosinophils and neutrophils. It is easy to mistake one polylobar nucleus for multiple nuclei, which may seriously interfere with the classification and counting of leukocytes. Therefore, by analyzing large numbers of blood leukocyte images, a segmentation method of blood leukocyte polylobar nucleus based on morphology is proposed. Compared with the image segmentation method based on geometric deformable model and genetic algorithm, the proposed method has faster convergence speed and shorter time consumption; compared with the particle counting method based on the principle of electrical impedance, it does not destroy the initial sample of blood and is easy to establish a database. Firstly, the leukocyte nuclei and platelets are segmented by using the difference between B component and G component of the leukocyte image. To remove platelets and obtain accurate leukocyte nuclei, the area threshold is used to filter out platelets because the area of every platelet is much smaller than that of any leukocyte nucleus. Due to the morphological [27] differences of the five types of blood leukocytes, such as the shape of nucleus and the size of nucleus, the image segmentation of leucocyte polylobar nuclei has achieved good segmentation results. After segmentation and judgment, the number of polylobar leukocytes can be accurately counted, which can be used in clinical medicine to provide the basis for the diagnosis of human health and reduce the workload of medical staff.

The article "A Polylobar Nucleus Identifying and Extracting Method for Leukocyte Counting" was published in 2021. Journal: Comput Math Methods Med.

## 2. The Main Characteristics and Classification of Leukocytes

Leukocyte is an important cell in the human body, which has the function of phagocytosis and immunity and maintains the normal operation of human body function. Generally, leukocytes are divided into monocytes, lymphocytes, basophils, eosinophils, and neutrophils. After Wright's staining, there are differences in their morphology, size, nucleus structure, cytoplasmic color, particle size, and polylobar nuclei.  Figure 1 is a typical image of leukocytes.

Figure 1(a) shows monocytes. In general, monocytes account for 3%~8% of leukocytes. The body diameter is generally 14~20 *μ*m, and the volume is the largest. The shapes of the monocytes are mostly irregular, spherical, or ellipsoid, and the cytoplasm is smaller. There are many small particles in the cytoplasm, which are light blue after Wright's staining, and some have vacuoles; the nucleus is blue purple after Wright's staining, with various shapes, including oval and horseshoe.  Figure 1(b) shows large lymphocytes. In general, lymphocytes account for 20%~40% of leukocytes. The body diameter of large lymphocytes is generally 10~20 *μ*m, and the shapes of lymphocytes are mostly spherical. After Wright staining, the nucleus is purplish red.  Figure 1(c) shows small lymphocytes. The body diameter of small lymphocytes is generally 6~9 *μ*m. The shapes of small lymphocytes are spherical or ellipsoidal, and the cytoplasm is smaller. In the case of small probability, there are pits. After Wright's staining, the nucleus is purplish red.  Figure 1(d) shows basophils. In general, basophils account for 0%~1% of leukocytes, which is the smallest type. The body diameter is generally 10~12 *μ*m, and the shapes of basophils are mostly spherical or quasispherical, with less cytoplasm. A small number of purple black basophilic granules are randomly attached to the basophilic bodies, which are light red after Wright's staining. Due to the presence of basophilic granules in the cytoplasm, light red holes usually appear after staining. The nucleus generally has no polylobar nucleus, and the nucleus is dark blue after staining. Figures 1(e) and 1(f) are eosinophils. In general, eosinophils account for 1%~5% of leukocytes, with a small proportion. The body diameter is generally 13~15 *μ*m, about twice the diameter of erythrocytes, and the shapes of eosinophils are mostly spherical. In Figure 1(e), there are many large eosinophils in the cytoplasm of rod-shaped eosinophils, which are light purplish red after Wright's staining and darker than neutrophils. The nucleus of the polylobar eosinophils in Figure 1(f) is usually two-lobed and “8” shaped. Figures 1(g) and 1(h) are neutrophils. In general, neutrophils account for 50%~70% of leukocytes, and the body diameter is generally 10~12 *μ*m, which is about 1.5 times of erythrocytes in diameter. The shapes of neutrophils are mostly spherical, and the cytoplasm is rich. After Wright's staining, the cytoplasm is generally light red or pink, and there are many small red particles evenly distributed. After staining, the nucleus is purplish, red, and curved petal shaped. The rod-shaped neutrophils in Figure 1(g) are immature leukocytes. The nucleus is slender, uniform in thickness, and mostly U-shaped. The polylobar neutrophil nucleus in Figure 1(h) is usually divided into 2 to 5 leaves, and there are three kinds of connections between the polylobar nuclei: filaments connected, overlapping with each other, and completely disconnected.

The article "A Polylobar Nucleus Identifying and Extracting Method for Leukocyte Counting" was published in 2021. Journal: Comput Math Methods Med.

From the five main characteristics of leukocytes, we can see that basophils, lymphocytes, and monocytes are mostly unilobar nuclei, while neutrophils and eosinophils have polylobar nuclei. In addition, neutrophils account for 50% to 70% of leukocytes, and it is easy to mistakenly divide one polylobar nucleus into multiple nuclei, which may cause misjudgments in the leukocyte count and cause medical accidents. Therefore, the accurate count of leukocytes is particularly critical, it should be an accurate segmentation of leukocytes, and then, count to determine.

## 3. Division of Leukocytes

### 3.1. RGB Color Space Model

The RGB color space model is based on the Cartesian coordinate system. In the RGB model, each color appears in the primary color spectrum components of red, green, and blue. According to the principle of three primary colors, the amount of light is expressed in primary color light units, as shown in formula (1). Therefore, in RGB color space, any color can be generated by superimposing and mixing three colors of red, green, and blue in different proportions. Each scale coefficient is different, resulting in different colors, such as blue is (0,0,255), then the red green scale coefficient is 0.

(1) $$\begin{array}{c} I_{C}=I_{R}\overset{⟶}{R}+I_{G}\overset{⟶}{G}+I_{B}\overset{⟶}{B}. \end{array}$$

RGB color space can be represented by a cube, as shown in Figure 2(a). Red, green, and blue represent three axes, corresponding to *x*, *y*, and *z* axes, respectively. The coordinate value range of each axis is usually 0~255. Along the main diagonal, from black to white, the gray level is getting higher and higher, and the total number of colors is(2^8^)^3^ = 16777216.

The article "A Polylobar Nucleus Identifying and Extracting Method for Leukocyte Counting" was published in 2021. Journal: Comput Math Methods Med.

Figure 2(b) shows the RGB color model. When the red, green, and blue components are all 0, they are at the origin, and the color mixture is superimposed as black; when the red, green, and blue components are all 255, the color mixture is superimposed as white; in addition, the other three diagonal vertices are represented as magenta (255, 0, 255), cyan (0, 255, 255), and yellow (255, 255, 0), respectively.

### 3.2. Analysis of the Segmentation Method Based on Otsu Threshold and Area Threshold

Yi-Ping Yang of our laboratory pointed out that the B-component and G-component images of leukocytes have obvious differences under different pH values and different light distributions [28].  Figure 3(a) shows the high-power microscopic image of leukocytes, Figures 3(b) and 3(c) show the G component and B component of Figure 3(a), respectively. By comparison, it can be seen that the difference between the white nucleus and platelet area is large, as shown in Figure 3(d). At the same time, the histogram analysis of Figures 3(b)–3(d), respectively, corresponds to Figures 3(e)–3(g).

In Figure 3(d), there is a gray value of *T*_1_, which can clearly distinguish the background area, erythrocyte area, and leukocyte cytoplasm area from the blood leukocyte nucleus area and platelet area. Therefore, the Otsu method is considered to select the optimal segmentation threshold which is more suitable for obtaining the leukocyte nucleus in the empirical threshold, as shown in Figure 4(a).

The leukocyte nucleus and platelet regions are obtained by the above method, and then, the area threshold is used to segment the leukocyte nucleus area. The area threshold segmentation is similar to the gray threshold segmentation. Through a large number of experiments, the experimental data is obtained, and the minimum value of the leukocyte nucleus area is calculated and set as the empirical threshold. The area threshold segmentation method is as follows: let *S* be the threshold area, *f*(*x*, *y*) be the initial binary image, and *g*(*x*, *y*) be the binary image after removal.

(2) $$\begin{array}{c} g\left(x,y\right)=\left\{\begin{array}{cc} 1 & f\left(x,y\right)\geq S,\\ 0 & f\left(x,y\right)<S. \end{array}\right. \end{array}$$

If the value of *f*(*x*, *y*) is greater than or equal to *S*, the value of *g*(*x*, *y*) is 1; otherwise, the value of  *g*(*x*, *y*) is 0. The empirical threshold based on the area threshold segmentation method can segment the area of leukocyte nucleus and platelets. The area with *g*(*x*, *y*) value 1 is the area of the leukocyte nucleus to be retained, and the area with *g*(*x*, *y*) value 0 is the area of the platelet to be removed, as shown in Figure 4(b).

The article "A Polylobar Nucleus Identifying and Extracting Method for Leukocyte Counting" was published in 2021. Journal: Comput Math Methods Med.

After segmentation of the leukocyte nucleus region, the segmentation edges are relatively complete. To verify whether the segmentation result is oversegmented or undersegmented, the segmented monochromatic binary image is stained first and, then, superimposed on the original image to observe the surrounding edges. As shown in Figure 5, where Figure 5(a) is a microscopic image of leukocytes, Figure 5(b) is the stained image, and the segmentation of Figures 5(a) and 5(c) is the effect superposition diagram of Figures 5(a) and 5(b).

Due to the presence of polylobar nuclei in neutrophils and eosinophils, after segmentation, there are two kinds of nucleus items: connected or disconnected, as shown in Figure 6. If the disconnected polylobar nucleus leukocytes are not judged, it is easy to mistake a single polylobar nucleus leukocyte as multiple unilobar nucleus leukocytes, leading to deviations in the leukocyte count.

## 4. Judgment of the Leukocyte Nucleus

### 4.1. Morphological Characteristic Parameters of Blood Leukocytes Based on Morphology

Because the five types of blood leukocytes have different appearances, they can be distinguished based on the morphological characteristics of leukocytes. The morphological characteristics include area, eccentricity, rectangularity, and ellipticity. The analysis of a large number of experimental data proved that using the five typical parameters of leukocyte nucleus area, leukocyte nucleus circumscribed rectangle plumpness, leukocyte nucleus circumscribed rectangle length-width ratio, leukocyte nucleus circumscribed ellipse plumpness, and leukocyte nucleus centrifugation rate can classify polylobar leukocytes and unilobar leukocytes.

The area of the leukocyte nucleus is a typical feature. Generally, the area is calculated by calculating the sum of pixels within the boundary of the area. Let *A* be the sum of pixels in the nucleus region of leukocytes; the calculation formula is as follows:

(3) $$\begin{array}{c} A=\sum \begin{array}{c} M\\ x=1 \end{array}\sum \begin{array}{c} N\\ y=1 \end{array}f\left(x,y\right). \end{array}$$

If the pixel (*x*, *y*) belongs to the nucleus area, then *f*(*x*, *y*) is assigned to 1; otherwise, *f*(*x*, *y*) is assigned to 0, that is, the area is equal to the sum of pixels in the nucleus area.

The fullness of the leukocyte nucleus can be measured by circumscribing a rectangular template. At this time, the fullness is the ratio of the area of the leukocyte nucleus to the area of the circumscribed rectangle, and its calculation formula is as follows:

(4) $$\begin{array}{c} P_{1}=A/a_{1}b_{1}, \end{array}$$

where *a*_1_ is the length of the circumscribed rectangle and *b*_1_ is the width of the circumscribed rectangle, that is, the ratio of the area of the nucleus to the area of the circumscribed rectangle is used to measure the plumpness of the leukocyte nucleus.

The article "A Polylobar Nucleus Identifying and Extracting Method for Leukocyte Counting" was published in 2021. Journal: Comput Math Methods Med.

The aspect ratio of the circumscribed rectangle can be used to measure the posture of the nucleus:

(5) $$\begin{array}{c} s=\frac{b_{1}}{a_{1}}. \end{array}$$

*s* approaching 1 means that the shape of the nucleus is round and the posture has no obvious trend, or the shape of the nucleus is shown as a bar and the posture tends to a 45-degree angle; *s* approaches 0 or *s* is much greater than 1 represents the appearance of the nucleus thin strips and their posture tends to be upright or lying down.

The above method measures the plumpness of the leukocyte nuclei by the circumscribed rectangles, and it can also be measured by the circumscribed ellipse template. At this time, the plumpness is the ratio of the area of the leukocyte nucleus to the area of a circumscribed ellipse. The calculation formula is as follows:

(6) $$\begin{array}{c} P_{2}=A/\pi a_{2}b_{2}, \end{array}$$

where *a*_2_ is the long axis of the circumscribed ellipse of the leukocyte nucleus and *b*_2_ is the short axis of the circumscribed ellipse of the leukocyte nucleus. The major axis and minor axis of the ellipse are unique, which can not only measure the plumpness of the leukocyte nucleus but also show the posture characteristics of the leukocyte nucleus from the direction of its major axis.

The eccentricity of the ellipse circumscribed by the leukocyte nucleus is defined as the ratio of the distance from the moving point to the left (right) focal point and the distance from the moving point to the left (right) guideline. The eccentricity can measure the flatness of the graph and is represented by *e*. The calculation formula is as follows:

(7) $$\begin{array}{c} e=\sqrt{a_{2}^{2}-b_{2}^{2}}/a_{2}. \end{array}$$

The value of *e* is between 0 and 1. The value of *e* tends to 0, which means that the graph tends to a circle, and the value of *e* tends to 1, which means that the graph tends to a flat ellipse.

According to the above five morphological characteristics, the nucleus of the polylobar nucleus leukocyte is judged. The algorithm flow is as follows:

1. Read a microscopic image of leukocytes, and use the above algorithm to segment the image of the leukocyte nucleus
2. After a large number of experimental data analysis and summaries, if the centrifugation rate of the leukocyte nucleus is greater than the corresponding empirical threshold *X*_1_ and the degree of ellipticity of the leukocyte nucleus is less than the corresponding empirical threshold *X*_2_, it may be judged as polylobar leukocytes, including neutrophils and eosinophils; otherwise, proceed to the next step
3. If the fullness of the circumscribed rectangle of the leukocyte nucleus is less than the corresponding empirical threshold *X*_3_, and the aspect ratio of the circumscribed rectangle is less than the corresponding empirical threshold *X*_4_, it may be judged as a polylobar nucleus leukocyte; otherwise, proceed to the next step
4. If the leukocyte nucleus area is less than the corresponding empirical threshold *X*_5_, it is judged as a polylobar nucleus leukocyte; otherwise, it is a unilobar nucleus leukocyte

The algorithm flow chart of the above operation steps is shown in Figure 7.

The article "A Polylobar Nucleus Identifying and Extracting Method for Leukocyte Counting" was published in 2021. Journal: Comput Math Methods Med.

### 4.2. Leukocyte Nucleus Extraction

The proportion of various types of leukocytes is an important indicator for medical staff to judge whether the human body is healthy or not. If a leukocyte is counted repeatedly, the proportion of various types of leukocytes will change, which may cause misdiagnosis. After the determination of leucocytes in the polylobar nucleus, it is found that the neutrophil nucleus will be completely disconnected from each lobule, as shown in Figure 8. This complete disconnection is due to the fact that when shooting under a microscope, it cannot be photographed or observed by human eyes. In reality, there are mitotic connections to provide nutrients between these leaves to the polylobar nucleus. If we do not judge the disconnection, it will lead to repeated counting of leucocytes. Therefore, we need to determine whether the segmented leaves belong to the same nucleus. The specific steps are as follows.

Suppose there are *n* regions in an image that are segmented, as shown in Figure 9:

1. Mark connected area
2. Use Canny edge detection operator to realize edge detection on the area in the image
3. Calculate the minimal distance between the current connected domain and the remaining connected domains, and connect
4. To fill the connected area after the connection
5. Repeat step 1–4 until all leaves are processed

After determining the number of leukocytes, count them according to the number of connected areas. Set the total number as *T*, neutrophils as *T*_*N*_, eosinophils as *T*_*E*_, basophils as *T*_*B*_, monocytes as *T*_*M*_, and lymphocytes as *T*_*L*_. If the total number of five types of leukocytes is greater than *T*, stop counting.

The article "A Polylobar Nucleus Identifying and Extracting Method for Leukocyte Counting" was published in 2021. Journal: Comput Math Methods Med.

## 5. Experimental Results and Analysis

### 5.1. Judgment Results and Analysis of Leukocyte Count

To verify this method, experiments are carried out on 8600 microscopic images of blood leukocytes under different dyeing conditions and different lighting conditions, and it is found that there are four cases which may lead to misjudgment.

**Case 1 .**

In a blood leukocyte microscopic image, there is only a single polylobar nucleus. The minimal distance connection is used many times to determine the connected domain and count, as shown in Figure 10.

**Case 2 .**

In a blood leukocyte microscopic image, basophils, monocytes, or lymphocytes exist at the same time, and the distance is close. Based on the nucleus area and nucleus circumscribed ellipse fullness degree, the connected domain is determined and counted, as shown in Figure 11.

**Case 3 .**

In a blood leukocyte microscopic image, the unilobar nucleus and the polylobar nucleus exist at the same time, and the distance is similar. Based on the nucleus area, the degree of ellipticity, and the minimal distance, the connected domain is found and counted, as shown in Figure 12.

**Case 4 .**

In a blood leukocyte microscopic image, two polylobar nuclei exist at the same time, and the distance is similar. Based on the cytoplasmic fullness and the minimal distance, the connected domain is found and counted, as shown in Figure 13.

From the results of experimental data, it can be concluded that the proposed method can realize the accurate count and determination of blood leukocytes, whether it is a polylobar nucleus leukocyte, or multiple polylobar leukocytes, or a unilobar nucleus leukocyte, which reflects the potential clinical application value.

### 5.2. Results and Analysis of Blood Leukocyte Segmentation Accuracy

To verify the accuracy of the segmentation accuracy of this method, experiments are carried out on microscopic images of blood leukocytes under different dyeing conditions and different lighting conditions, and the four cases of blood leukocytes that are prone to misjudgment are put together with other blood leukocytes for segmentation processing.  Figure 14 is the random processing of 30 groups of experimental results.

In Figure 14, No.1 is the segmentation accuracy result of the single polylobar leukocyte mentioned in Case 1, No.7 is the segmentation accuracy result of the single unilobar leukocyte mentioned in Case 2, No.20 is the segmentation accuracy result of the one polylobar leukocyte and one unilobar leukocyte mentioned in Case 3, and No.6 is the segmentation accuracy result of two polylobar leukocytes mentioned in Case 4.

It can be seen from the high-magnification microscopic image of leukocytes, the image after leukocyte nucleus staining, and the image overlay effect that the proposed method achieves accurate segmentation without oversegmentation and undersegmentation, to identify and extract the leukocytes from the polylobar nuclei. The experimental results show the high-precision characteristics of the proposed method.

The article "A Polylobar Nucleus Identifying and Extracting Method for Leukocyte Counting" was published in 2021. Journal: Comput Math Methods Med.

Yang et al. proposed a leukocyte segmentation method based on the Otsu method, randomly selected 300 leukocyte microscopic images for experiments, and compared the proposed method with Yang's method for the segmentation rate of leukocyte nuclei. The experimental results are shown in Table 1. According to statistics, the microscopic images of 300 leukocytes used in the experiment were 113 neutrophils, 36 eosinophils, 18 basophils, 69 monocytes, and 64 lymphocytes.

It can be seen from the experimental results that the experimental results of the two methods perform well. The average segmentation accuracy of the proposed method is 98.3%, which is higher than that of Yang's method (96.6%). Since basophils are produced under severe human diseases, the number of samples of this type of white blood cells is relatively small. Although the number of samples of this type of leukocyte is very small during the experiment, the segmentation accuracy has reached 94.4%, and the stability of the algorithm is also good. Experimental results show that this method has high accuracy and stability.

In order to ensure the fairness of the experiment, the samples used are all original samples without any processing. The time-consuming of the proposed method is 3 ms. Compared with the image segmentation algorithm of the genetic algorithm, the time-consuming is shorter.

Through a large number of experimental results, it can be known that the polylobar nuclear leukocyte segmentation method using Otsu and area threshold has good applicability, stability, and segmentation accuracy.

## 6. Conclusion

In this paper, leukocytes under different staining conditions and different lighting conditions are accurately segmented by the difference between the B component and the G component in color space, the Otsu threshold method, and the area threshold method. At the same time, based on the morphological method and the minimal distance method, the connection and number of polylobar nucleus leukocytes are determined. By using the proposed method, we can accurately count the polylobar leukocytes which are completely disconnected and will not count them into multiple leukocytes by mistake. It can also reduce the counting error caused by manual microscopic test and reduce the workload of medical staff. Of course, the proposed method is based on microscopic imaging. When all the leaves from the same polylobar nuclear leukocyte are overlapped at a certain shooting angle, this method may be limited. Fortunately, a large number of experiments show that this situation rarely occurs because the leukocyte image is taken on the deposited blood smear. The experiment proves the feasibility and practicability of the proposed method, which provides a solid foundation for the accurate count of blood leukocytes.

The article "A Polylobar Nucleus Identifying and Extracting Method for Leukocyte Counting" was published in 2021. Journal: Comput Math Methods Med.

## Figures and Tables

**Figure 1:** Microscopic images of five types of blood leukocytes.

**Figure 2:** RGB color model.

**Figure 3:** Components and histogram of leukocyte high power microscopic image.

**Figure 4:** Experimental results processing diagram.

**Figure 5:** Leukocyte microscopic image and superposition effect diagram.

**Figure 6:** The leukocytes of two kinds of polylobar nuclei after segmentation.

**Figure 7:** Flow chart of classification and determination algorithm for polylobar leukocytes.

**Figure 8:** The connection of leukocytes in the polylobar nucleus.

**Figure 9:** Segmentation results of polylobar nucleus leukocytes.

**Figure 10:** Single polylobar nucleus leukocyte count determination results.

**Figure 11:** Two unilobar nucleus leukocytes count determination results.

**Figure 12:** Results of counting one unilobar nucleus leukocyte and one polylobar nucleus leukocyte.

**Figure 13:** Results of two polylobar nuclei leukocyte counts.

**Figure 14:** The results of segmentation of leukocytes by this method.

**Table 1:** Segmentation accuracy of the five types of leukocytes.

Leukocyte class	Number of samples	Segmentation method			
		Yang's method		Proposed method	
		Result of segment	Accuracy (%)	Result of segment	Accuracy (%)
Neutrophil	113	112	99.1%	112	99.1%
Eosinophil	36	34	94.4%	35	97.2%
Basophil	18	16	88.8%	17	94.4%
Monocyte	69	67	97.1%	68	98.5%
Lymphocyte	64	61	95.3%	63	98.4%
Total	300	290	96.6%	295	98.3%

## Data Availability

The data that support the findings of this study are available from the corresponding author upon reasonable request.
